# Assessing the Relationship between Resource Misallocation and Total Factor Productivity Based on Artificial Neural Network

**DOI:** 10.1155/2022/5148879

**Published:** 2022-06-17

**Authors:** Weiwei Zhang, Lan Bo, Shengqiang Zhang, Yuan Wang

**Affiliations:** Sunwah International Business School, Liaoning University, Shenyang 110136, China

## Abstract

For interpretation of China's economy, total factor productivity is considered as one of the crucial aspects which is generally dependent on innovation in technologies especially those driven by both scientific research and efficiency of the methodology or process which is dedicated for the allocation of numerous resources available, among enterprises. It is important to note that various factors, which are either directly or indirectly involved, to cause misallocation of the resources to the enterprises, are overly complex. Therefore, an affective mechanism is needed to be realized which is capable of resolving these issues with the available resources and infrastructures. In this paper, we have focused on the construction or development of an artificial neutral network (ANN) based evaluation model to study the impact of resource misallocation on total factor productivity. Likewise, we have conducted a counterfactual experiment, i.e., simulation only, to thoroughly examine the relationship between two very important factors, that is, (i) resource misallocation and (ii) total factor productivity. To do this, we are aiming at investigating the growth potential of total factor productivity when there is no resource misallocation. After comparing 8 industries in different regions, we conclude that the contribution of capital and labor distortion to total factor productivity is the highest in the eastern region of China with −0.036 and 0.065, respectively, followed by the northeast, central, and western regions. In the experiment, China's total factor productivity growth potential could reach 1.1296, if there is no resource misallocation. The results in this paper would shed some lights on the paths to improve resource allocation efficiency and total factor productivity.

## 1. Introduction

Manufacturing is the process of converting raw materials or parts into completed things using tools, human labor, equipment, and chemical processes. Manufacturing enables companies to sell completed goods for more than the cost of the raw materials required. Large-scale manufacturing enables the mass production of items employing assembly line procedures and innovative technology as primary assets. Manufacturers may take advantage of economies of scale by using efficient manufacturing processes to produce more units for less money. In the context of the “new normal” of the economy, China's manufacturing industry has long relied on resource input to achieve economic growth and changing the economic growth mode had become the necessity to implement the strategy of strengthening the country. The 2015 Chinese government work report first mentioned the concept of total factor productivity (TFP) improvement and proposed the fact that total factor productivity improvement is the major driving force for sustainable economic growth under the background of the “new normal” and it is necessary to rationally allocate resources and upgrade the manufacturing structure. In this regard, this paper focuses on the improper allocation of manufacturing resources and its impact on TFP. Resource misallocation is the performance of resources not being reasonably and effectively allocated. High-quality economic development in countries and regions could be promoted by high TFP. However, the current situation of resource misallocation in China limits the TFP improvement.

The allocation process of resource, i.e., optimality in this case, is a fundamental topic in economics. In most cases, effective resource flow increases productivity, while resource misallocation can stymie economic progress. Resource depletion has become a barrier to the improvement of market companies as a developing country in transition. Furthermore, the current resource distribution model inhibits the flow of resources, causing the entire sector to weaken. Improper resource allocation results in decreased production efficiency and excessive losses, threatening China's economy long-term viability.

Therefore, to resolve this issue, an empirical research on the misallocation of manufacturing resources and changes in total factor productivity of listed companies is carried out in this paper, which would shed light on the paths to improve resource allocation efficiency and total factor productivity. Furthermore, artificial neural network-enabled model is utilized for this purpose which has achieved maximum accuracy.

The rest of the paper is organized as follows.

In the coming section, innovations along with detailed description of the existing studies are reported with supportive literature review. In Section 3, the proposed artificial neural network experimental evaluation model and its construction mechanism are described. Moreover, various sections of this model and working procedures are described further. Various results collected to the proposed model are compared with the existing models and presented in Section 4 along with justifiable discussion. At the end, concluding remarks are given.

## 2. Literature Review and Innovations

The research on determining the wealth of a country (region) has developed from the accumulation of capital and labor force in a country (region) to the improvement of total factor productivity (TFP) (Hsieh and Klenow) [1]. The weighted average of inputs, such as labor and capital, is used to compute total factor productivity (TFP). It denotes actual production growth that outpaces increase in labor and capital inputs. Understanding the development differences between different countries (regions) from the perspective of resource misallocation is one of the fastest-growing fields in the research on economic growth in recent 10 years (Syverson) [2]. Given capital and labor input, the way by which they are allocated among different sectors determines the productivity level of an economy. In the long run, the optimal resource allocation will maximize output and social welfare, while resource misallocation will lead to a lower level of TFP. Restuccia and Rogerson [3] as well as Bartelsman et al. [4] tried to prove theoretically and empirically that the resource mismatch between developing and developed countries explains the substantive part of the TFP difference between developing and developed countries. From the existing research, the measurement of national or regional economic growth level by TFP has been recognized by most researches, and there is basically a consensus that resource misallocation will reduce the TFP of a country or region (Luo et al.) [5–8].

As the largest developing country and transitional economy, resource misallocation problem in China has attracted great attention. The relevant literature is mainly carried out by estimating the TFP level of enterprises and measuring the degree of resource misallocation with a series of TFP decomposition techniques such as TFP dispersion and OP covariance (Färe et al.) [9, 10]. These studies have found the different degrees of resource misallocation among Chinese industrial enterprises（Nie et al.) [11–13]. From another perspective，Hsieh and Klenow [14] tried to establish a mathematical model about the relationship between resource misallocation and TFP and established a reference frame for data calibration to solve the problem of “how much efficiency will be improved if the distortion of resource allocation disappears.” By using a monopoly competition model and relevant data, they found that if the capital and labor force of China and India are reconfigured to reach the same level of marginal output as the United States, the TFP of manufacturing industry in the two countries will increase by 30%∼50% and 40%∼60%, respectively. Brandt et al. [15] used the provincial level data of China's nonagricultural sector from 1985 to 2007 to focus on the TFP loss caused by the distorted allocation of capital and labor factors in different regions and between different ownership systems. The results showed that between 1985 and 2007 the resource mismatch reduced the TFP of the nonagricultural sector by 30%, of which the mismatch between provinces and within provinces contributed half. Tang et al. [16] used mitigation-based poor model measures to analyze the efficiency of environmental regulations and used data envelopes to divide total factor productivity. The results show that TFP has an obvious “clustering” effect in China.

This paper examines the link between total factor productivity and resource misallocation in several industries, as well as the relationship between total factor productivity and resource allocation, and concludes that better resource allocation improves total factor productivity. The artificial neural network regression model is utilized to measure in this study, and the general regression model may be estimated with the neural network. However, there is no report of using a neural network to do probability calculations. In a probabilistic sense, the stochastic frontier model adds a frontier (data envelope) to the normal regression. After the normal regression, this frontier function is calculated. Based on this feature, this paper constructs a branched neural network that implements TFP measurement using a probabilistic frontier model. All calculation procedures are calculated by programming included in the DASC system. The concept of bifurcation neural network is proposed, which enriches the theory of neural network.

## 3. Construction of the Artificial Neural Network Experimental Evaluation Model

Artificial neural networks (ANNs) and simulated neural networks (SNNs) are types of neural networks used in deep learning techniques. The human brain inspired its name and structure, which mimics how organic neurons communicate with one another. A node layer consists of an input layer, one or more hidden layers, and an output layer in artificial neural networks. Each node, or artificial neuron, is connected to the next and has a weight and threshold associated with it. If a node's output exceeds a certain threshold, the node is activated, and data is sent to the network's next tier. Aside from that, no data is carried on to the network's next tier.

### 3.1. Calculation of Mismatch Indicators for Provinces

#### 3.1.1. Capital Margin and Labor Margin

Cobb-Douglas production function method is selected to calculate the degree of resource misallocation. The Cobb-Douglas production function can generally be expressed in the following traditional form:

(1) $$\begin{array}{c} Y=AK^{a}L^{b}. \end{array}$$

In formula (1), *Y* represents output, capital is represented by *K*, and labor is represented by *L*. a and *b*, respectively, represent the output elasticity of capital and labor. When the scale effect is constant, *a* + *b* = 1. *K*_*it*_ and *I*_*it*_, respectively, represent the capital and labor input of *i* province in *t* period, and *K*_*it*_ is calculated by perpetual inventory method.

(2) $$\begin{array}{c} K_{it}=K_{it-1}\left(1-∆t\right)+I_{it}, \end{array}$$

where *K*_*it*_ represents the current capital stock, *K*_*it*−1_ represents the remaining capital stock of the previous period, and the earlier the base year is selected, the smaller the influence of the error of the capital stock of the base year on the subsequent years becomes (Huber) [17]. Combined with the availability of data, this paper selects 1952 as the standard base period, the fixed capital formation in 1952 divided by 10% as the initial capital stock, and Δ*t* represents the economic depreciation rate, which is generally 9.6%. Further, capital marginal product and labor marginal product are obtained.

(3) $$\begin{array}{c} {\text{MPk}}_{it}=\frac{\text{dY}}{\text{d}K},\\ {\text{MPl}}_{it}=\frac{\text{dY}}{\text{d}L}, \end{array}$$

where *MPk*_*it*_ represents the capital marginal product of *i* province in *t* period, and MPl_it_ represents the labor marginal product of *i* province in *t* period. Comparing marginal product with the actual price has important economic significance.

(4) $$\begin{array}{c} r=\frac{DE+OS+NT\left(DE+OS\right)}{\left(WL+DE+OS\right)k_{it}}, \end{array}$$

where *r* is the actual reported turnover of capital elements in the market, representing the output of capital elements, DE is the depreciation of fixed assets, OS is the operating surplus, NT is the net production tax, WL is the actual salaries of capital factors, and *k*_*it*_ is the capital input.

(5) $$\begin{array}{c} \text{dis}k_{it}=\frac{{\text{MPk}}_{it}}{r}\\ \text{dis}l_{it}=\frac{{\text{MPl}}_{it}}{w}, \end{array}$$

where dis*k*_*it*_ and dis*l*_*it*_ are the absolute mismatch indicates of capital and labor, respectively, and *w* represents the actual salaries of labor factors in the market. When dis*k*_*it*_ > 1, capital factors are underestimated and the price of capital factors is negatively distorted (Reiss et al.) [18]. When dis*k*_*it*_ = 1, the capital factor price is equal to the capital marginal product, and there is no distortion of the capital factor price. When dis*k*_*it*_ < 1, the capital factor is overestimated, the price of capital factor is distorted positively, and the labor factor is the same.

#### 3.1.2. Time-Varying Elastic Production Function

The link between production output and production inputs is modelled by a Cobb-Douglas production function (factors). It is used to measure technical progress in manufacturing processes and determine input-output ratios for efficient production. This model is based on the assumption that is not in line with economic reality; that is, the output elasticities *a* and *b* of the capital and labor factors are assumed to be fixed constants. In the logarithmic form of the time-varying elastic production function, the output elasticities are replaced by nonparametric smoothing functions *a(t)* and *b(t)*. The output elasticity at this time is a function of time *t*, and the production function is also a time-varying elastic production function. The function at this time is more in line with the economic reality that factor prices and quantities change over time. The time-varying elastic production function model can be expressed as

(6) $$\begin{array}{c} \text{ln}Y_{t}=\sum_{i=1}^{n}e_{i}X_{i}+a\left(t\right)\text{ln}K_{t}+b\left(t\right)\text{ln}L_{t}+u_{t}. \end{array}$$

In (6), *e*_*i*_ represents an unknown parameter, *X* is a controllable variable, *X*_i_ is a variety of indicators to measure the skill level, *e*_*i*_*X*_*i*_ is a set of controllable variables *X*, that is, a linear combination, and *K*_t_ represents the technical level. This is the time-varying elastic production function that improves the neutral skill level assumption. At present, the application of the time-varying elastic production function in the research method of resource misallocation is still in the stage of exploration and development (Huber) [17].

#### 3.1.3. Profit Function Method

The profit function method is more focused on examining the market situation when the enterprise's profit is maximized by derivation of the production function. The formula is as follows:

(7) $$\begin{array}{c} u_{i}^{*}=\varphi_{i}u_{i}q^{*}=\varphi q. \end{array}$$

In (7), *u*_*i*_^*∗*^ and *u*_*i*_ are the equilibrium price and market price of production factors, respectively, and *q*^*∗*^ and *q* are the equilibrium price and market price of the product, respectively. In the absence of trade friction, the equilibrium price is the same as the market price, so they are equal. By introducing methods such as the profit share function of the enterprise, the value of *φ*_*i*_ can be estimated. When *φ*_*i*_ = 1, there is no mismatch of resources. The corporate profit function commonly used in research is

(8) $$\begin{array}{c} \prod_{j}=p_{k}AK^{a}L^{b}-\left(1+t_{k_{j}}\right)k_{j}-\left(1+t_{L_{j}}\right)L_{j}. \end{array}$$

In (8), *t*_*k*_*j*__ and *t*_*L*_*j*__ represent the capital factor distortion tax and labor factor distortion tax (mismatch coefficient) caused by resource misallocation, respectively. The price of a factor of production multiplied by (1 + *t*_*k*_*j*__) or (1 + *t*_*L*_*j*__) represents the market equilibrium price of the factor of production. The pursuit of profit maximization by an enterprise can be represented by the first-order condition of the profit function. The resource misallocation of capital factors and labor factors is, respectively, expressed as follows:

(9) $$\begin{array}{c} r\left(1+t_{k_{j}}\right)=\frac{PY_{j}a}{K_{j}},\\ w\left(1+t_{L_{j}}\right)=\frac{PY_{j}b}{L_{j}}. \end{array}$$

In (9), it is also possible to estimate the overall mismatch index of the economy and the extent to which resource misallocation affects TFP.

### 3.2. Resource Misallocation and TFP Indicators in China

Suppose that there is an industry *i* in the real economy and use the two elements of capital *K*_i_ and labor *L*_i_ to represent different products. Under free trade, the prices of capital and labor are *r* and *w*, respectively, but the prices actually paid are *(1* *+* *t*_*Ki*_*)r* and *(1* *+* *t*_*Li*_*)w*. Due to different products in different industries, even if the distortion tax rate is 0, the product price *P*_i_ may be different. Because the firm is a price taker and uses a constant-volume production function of relative size, the industry in the model can be replaced by a representative firm (Yeferny et al.) [19]. In this section, *Y*_*i*_ is output, *A*_*i*_ is TFP, and *a*_*i*_ is capital share. The first-order conditions for the firm's output maximization problem are as follows:

(10) $$\begin{array}{c} \frac{a_{i}P_{i}Y_{i}}{K_{i}}=\left(1+t_{k_{i}}\right)r, \end{array}$$

(11) $$\begin{array}{c} \frac{\left(1-a_{i}\right)P_{i}Y_{i}}{K_{i}}=\left(1+t_{L_{i}}\right)w. \end{array}$$

By combining (10) and (11), we can define the competitive equilibrium, given TFP and distorting tax rates {*A*_i_, *t*_Ki_, *t*_Li_} for each industry, as well as total factor stock K and labor *L*, output, capital, labor, and goods (Kim et al.) [20]. The prices {*Y*_i_, *K*_i_, *L*_i_, *P*_i_} of various industries that satisfy the conditions constitute a competitive equilibrium. The expression for *K*_i_ can be given:

(12) $$\begin{array}{c} K_{i}=\frac{{\bar{s}}_{i}a_{i}}{\bar{a}}{\bar{p}}_{Ki}K, \end{array}$$

where ${\bar{s}}_{i}$ is the share of industry output *P*_*i*_*Y*_*i*_/*Y* and the overline indicates that this variable is related to the specific form of the aggregate function. $\bar{a}$ is the weighted average of $\sum_{i}{\bar{s}}_{i}a_{i}$ of each industry's capital share, and ${\bar{p}}_{Ki}$ measures the relative distortion of industry *i*:

(13) $$\begin{array}{c} {\bar{p}}_{Ki}=\frac{P_{Ki}}{\sum_{j}\left({\bar{s}}_{j}a_{j}/\bar{a}\right)P_{Kj}},\\ P_{Ki}=\frac{1}{1+t_{k_{i}}}. \end{array}$$

By decomposing the total output, the resource misallocation loss of the entire TFP can be seen intuitively. First, the sum function is expanded logarithmically.

(14) $$\begin{array}{c} \text{ln}Y=\sum_{i}\frac{\partial \text{ln}Y}{\partial \text{ln}Y_{i}}\text{ln}Y_{i},\\ =\sum_{i}{\bar{s}}_{i}\text{ln}Y_{i}. \end{array}$$

The Solow residual method is also known as the production function method because it improves factor productivity (Lingfors et al.) [21].

(15) $$\begin{array}{c} \text{TFP}=\sum_{i}{\bar{s}}_{i}\text{ln}\left(A_{i}\right)+\sum_{i}{\bar{s}}_{i}\left(a_{i}\text{ln}{\bar{p}}_{Ki}+\left(1-a_{i}\right)\text{ln}{\bar{p}}_{Li}\right). \end{array}$$

The entire TFP can be divided into two parts. The former is the weighted average of the total factor productivity of each industry, and the latter can be defined as the loss of resource allocation efficiency caused by the distortion of differences among industries. The methodological advantage of (14) is that the divergence between capital and labor can be separated and compared directly.

(16) $$\begin{array}{c} AL_{K}=\sum_{i}{\bar{s}}_{i}a_{i}\text{ln}{\bar{p}}_{Ki},AL_{L}\\ =\sum_{i}{\bar{s}}_{i}\left(1-a_{i}\right)\text{ln}{\bar{p}}_{Li}. \end{array}$$

This data source is from the “China Industrial Economic Statistical Yearbook,” and the time period is from 2010 to 2020. The main variables used in this paper are industrial added value, net fixed assets, total number of employees, total accounts payable for the current year, and industrial sales (Raynaud et al.) [22].  Table 1 shows the descriptive statistics of the main variables after processing outliers.

*K *_*i*_ data from 2010 to 2020 is shown in Figure 1. It includes the weighted average and capital income ratio of all industrial enterprises in the northeast, central, eastern, and western regions. The northeast region includes Inner Mongolia, Liaoning, Jilin, and Heilongjiang, the central region includes Shanxi, Anhui, Jiangxi, Henan, Hubei, and Hunan, and the eastern region includes Beijing, Tianjin, Hebei, Liaoning, Shanghai, Jiangsu, Zhejiang, and Fujian. The western region includes Guangxi, Chongqing, Sichuan, Guizhou, Yunnan, and Shanxi.

During the period from 2010 to 2020, the average capital income increased slightly with the growth rate slowing down after 2015. Before 2015, the proportion of capital income in the northeast region was higher than that in the central and western regions and was subsequently surpassed by the central region.

Figure 2 shows the misallocation of capital and labor in the industrial sector and the loss of production due to misallocation and changes in industrial resources from 2010 to 2020.

Here, labor-intensive and resource-intensive industry indicators are selected to represent the entire industry. As can be seen from Figure 2, resource misallocation has a great impact on total output (or TFP), which decreases by an average of 17.5%. From the perspective of time trend, it deteriorated before 2015 and improved after 2015, but there was little difference from year to year (Shen et al.) [23]. In addition, the change in labor mismatch is small, and the change in the total capital-labor mismatch efficiency is mainly due to the change in capital mismatch.

### 3.3. Artificial Neural Network

The human brain is the most efficient intelligent system in the world. The brilliant achievements of human development depend on the information processing ability, information storage ability, and learning ability of the human brain. Scientists continue to study the human brain, simulating the structure and operation of the human brain, hoping to find out the mystery of the human brain. During this period, the most famous artificial neural network (ANN) theory was born. It designed many different algorithms according to the main functions of the human brain and established a mathematical model that can specifically deal with problems in practice (Souza et al.) [24]. The artificial neural network algorithm has the advantages of high error tolerance rate for sample data, strong nonlinear mapping ability, self-adaptation, and self-organization and has the advantages of self-learning and strong generalization ability. It has been widely used in the forecasting of factors of production and achieved ideal results. The artificial neural network is composed of several different modules, and each module is composed of multiple simple elements that can deal with complex problems. This structure enables the neural network to have the basis for processing complex information.

The role of neurons in biology is to process the information burst from each adjacent cell through the dendrite and finally transmit it to other adjacent neurons through the axon. The neurons of the artificial neural network are obtained according to the simplified biological neuron network, as shown in Figure 3.

There are multiple signal points in the figure, each input signal corresponds to a connection weight *w*, and the sum of the product of the input *p* and the weight *w* plus *b* becomes the input of *f*(·) in the neuron. The input *p*_j_ in the network is represented as *P* = [p_1_, *p*_2_,…, *p*_r_]^T^, and the weight *w*_*j*_ in the network can be represented as *W* = [w_1_, *w*_2_,…, *w*_*r*_]; then, the output of this simple network model is

(17) $$\begin{array}{c} A=f\left(W*P+b\right)\\ =f\left(\sum_{j=1}^{r}w_{j}p_{j}+b\right). \end{array}$$

In (17), *b*, as the input to adjust the activation function, plays a great role in the flexible use of the activation function. Therefore, determining the type of activation function is an important part of building a neural network model. Common activation functions are as follows.

#### 3.3.1. Threshold Function

Through the threshold function, no matter what data is input, the final output is 0 or 1. *f*(·) is the unit step function, as shown in Figure 4. The relation of the threshold function is

(18) $$\begin{array}{c} A=f\left(W*P+b\right)\\ =\left\{\begin{array}{c} 1,W*P+b\geq 0,\\ 0,W*P+b<0. \end{array}\right. \end{array}$$

#### 3.3.2. Linear Type

This type of function directly outputs the value calculated by (18), that is, the sum of the weighted sum and the deviation, as shown in Figure 5:

(19) $$\begin{array}{c} A=f\left(W*P+b\right)\\ =W*P+b. \end{array}$$

#### 3.3.3. S-Type Function

The input value is compressed into the range (0, 1) using the logarithmic function or the hyperbolic tangent function. The logarithmic activation function is as (18):

(20) $$\begin{array}{c} f=\frac{1}{1+\text{exp}\left(-n\right)}. \end{array}$$

The hyperbolic tangent activation function is as (18):

(21) $$\begin{array}{c} f=\frac{1-\text{exp}\left(-2n\right)}{1+\text{exp}\left(-2n\right)}. \end{array}$$

The sigmoid function is the most commonly used activation function in neural networks and can provide a nonlinear mapping from input to output. Artificial neural networks use this feature to process large and small signals. Small-signal problems are solved in the mid-high gain region of the function, and large-signal processing is solved in the low-gain regions on both sides [25]. Whether the artificial neural network system is a nonlinear system depends on whether the excitation function of the neuron is a nonlinear function.

## 4. Counterfactual Simulation

### 4.1. Measurement of Total Factor Productivity by Artificial Neural Network

This paper chooses gross domestic product (GDP) at comparable prices as a measure of China's total output. The standard measure of the value added generated by the production of goods and services in a country during a certain period is the gross domestic product (GDP). As a result, it also accounts for the revenue generated by that production, as well as the overall amount spent on final products and services (less imports). The first reason is that this indicator can be obtained directly from relevant statistics, and the second reason is that GDP can reflect the economic scale and development level of a region. This paper uses GDP as the basic indicator to measure economic growth and converts it at the constant price at the initial year [26].

TFP analysis should strictly follow theoretical requirements and calculate labor input based on the “service flow” provided by each element over a period of time. Labor input depends not only on the amount of factor input, but also on factors such as factor utilization efficiency and factor quality. Under the adjustment of the market mechanism, labor remuneration can reasonably reflect changes in labor input. This paper uses the number of employees in China over the years as an indicator of labor input over the years [26].

Capital input is defined as the flow of capital services provided by the capital stock. Here, this paper uses capital stock as a measure of capital input. According to the TFP expression of (14), the results of calculating TFP are shown in Table 2.

A three-layer artificial neural network is used to analyze the index system of the National Science Medal Innovation Index, which was created using the MATLAB neural network toolkit. This research creates an artificial neural network model based on the index system. There are 21, 8, and 2 neurons in the input layer, hidden layer, and output layer, respectively. For a training step, the maximum number of epochs is 2000, the convergence error goal is 1e − 30, and the display interval is 10. The Levenberg-Marquardt optimization algorithm's mu dec is 0.2, the increase factor is 1.2, the maximum mu max is le − l5, and the performance function min grad's minimum gradient is 1e − 15.

The training sample data is the index data of some countries published by the European Scoreboard in 2010. This data set is input in this paper. After the network is initialized, the function trainlm is used to train the network 13 times. The sum of the squared errors of the network mes meets the requirement of convergence error goal = le − 30 (Chen) [27]. The error curves of the training samples are shown in Figure 6.

As can be seen from Table 3 and Figure 6, the artificial neural network has been trained 13 times, and the obtained results are in perfect agreement with the expected output. This proves the effectiveness of the artificial neural network model designed in this paper.

Aiming at some drawbacks of the commonly used methods for measuring the R&D input contribution rate, this paper uses the input-output table to measure TFP and then the R&D input contribution rate and studies the method. According to the method introduced in Section 3, using DASC software, and using the relevant economic statistics from 2010 to 2020 from the National Bureau of Statistics and the transformation of statistical methods, the scatter of TFP and R&D contribution rate in 2010–2020 can be obtained, as shown in Figure 7.

In order to analyze the compositional contribution of China's economic growth, this paper quantitatively analyzes the output contribution of capital input, labor input, and total factor productivity to GDP based on the results measured by the new method. In general, China's economic growth is mainly driven by investment growth, and capital investment drives economic growth, but the role of total factor productivity cannot be ignored. Since 2010, total factor productivity has not maintained rapid growth, but it has contributed to China's economic growth.

### 4.2. The Relationship between Resource Misallocation and TFP

According to the calculation method of resource misallocation in Section 3.1, this paper calculates the average resource misallocation degree of some provinces in China in 2020, as shown in Table 3. The regions selected in this paper are all provinces with relatively developed industries in China.

According to the impact of resource distortion changes on output (total TFP), it is easy to obtain the various industrial contributions of factor distortions to overall economic output (Wu et al.) [28]. The left side of Figure 8 shows the contribution of capital distortions to TFP, and the right side shows the contribution of labor distortions to TFP.

1–8 in the figure represent electrical machinery and equipment manufacturing, steel and metal smelting and rolling industry, chemical raw material and product manufacturing, computer communication and other electronic equipment manufacturing, transportation equipment manufacturing, and general equipment manufacturing (Shair et al.) [29]. Through these typical Chinese industries, this study shows the overall trend of industrial development and upgrading. On the whole, changes in enterprise productivity, adjustment of factor structure among enterprises, and entry and exit of enterprises have all contributed to the improvement of total factor productivity to varying degrees. But, for firms, the contribution rate of changes in productivity dominates.

### 4.3. The Impact of Resource Misallocation on TFP

The impact mechanism of resource misallocation on total factor productivity is as follows: in a completely free market economy environment, production factors such as labor and capital always flow to regions and enterprises with high productivity. Based on the law of diminishing marginal utility, as the scale of labor and capital increases, its factor productivity will decrease. Ultimately, it achieves the fact that all firms in the market have the same total factor productivity. In practice, the free flow of factors will always be limited to a certain extent, so that the marginal outputs of various resources are not equal in cross section. This leads to overallocation of resources in some regions and underallocation in others, i.e., resource misallocation.

Whether industrial transformation affects regional technical efficiency or technological progress through resource misallocation and whether it has formed economies of scale still need discussion in the current research. On the one hand, due to the incomplete flow of resources, the spatial distribution of production factors cannot satisfy the equal marginal output. That is, the output cannot be maximized under the current technology, thus reducing its technical efficiency [30]. On the other hand, enterprises in areas with abundant production resources and low cost of production resources will increase factor input as much as possible in order to maintain a certain output. Macroscopically, the crowding-out effect of industrial capital transfer on technological progress and technological efficiency hinders the technological progress and improvement of technological efficiency in regions. To maintain a certain output, enterprises in areas with scarce resources and high factor costs are more inclined to promote technological progress through technological research and development, so as to offset or reduce the negative impact of resource misallocation on production efficiency. Under normal circumstances, the transfer of labor-intensive, resource-intensive, and even high-pollution, high-consumption industries in China is also based on the advantages of relatively abundant production resources and lower production costs.

It can be seen from the regression results of the place of industrial transfer that industrial transfer still has a positive effect on total factor productivity and at the same time industrial transfer reduces the degree of resource misallocation in the place of transfer, but its transmission mechanism is still insignificant [31]. In a return to inheritance, industrial transfer reduces total factor productivity. And, in terms of the transmission mechanism of resource misallocation, industrial transfer increases the degree of resource misallocation, and resource misallocation reduces total factor productivity. Resource misallocation presents an obvious transmission mechanism. The result of the impact path is shown in Figure 9.

As far as industries are transferred, resource misallocation will make the local industry more competitive with laborers, thus forcing the upgrading of the industries in the transfer destination. Therefore, resource misallocation is positively correlated with industrial upgrades. After estimating the output elasticity of the production function, the price distortion of each factor in the subindustry can be obtained, and the productivity status of individual enterprises can be calculated. Next, this paper weights the productivity coefficients of individual firms to obtain the aggregate productivity of the six corresponding subsectors and calculates the gap between actual output and potential output.  Figure 10 shows the gap between the actual TFP level and potential TFP growth space of some industries in 2020.

As can be seen from the figure, the difference in TFP between the six representative subsectors is a maximum of 3-4 times. Different from the resource-labor-intensive industries selected before, the industries with a large volume in China are selected here to observe the overall industry situation in China. The TFP of “ferrous metal smelting and rolling processing industry” is the highest, because the industry requires high factor input growth rate and factor accumulation. However, the growth rate of “ferrous metal smelting and rolling processing industry” during the observation period was negative, and the potential growth space of TFP did not change much.

Relatively speaking, the resources of the transfer area are relatively scarce and the cost is relatively high, which basically conforms to the theoretical analysis. The resource misallocation affects the path regression results on TFP, as shown in Table 4.

## 5. Conclusion

In this paper, we have tried to explore the manufacturing resources of China especially from the various perspectives such as total factor productivity and mismatch. It calculates the price distortion coefficients for capital and labor factors, as well as individual and overall distortion coefficients, and then analyzes the relationship between factor price distortion coefficients, resource misallocation coefficients, and total factor productivity using an artificial neural network algorithm. TFP of various industries is estimated, as well as the trend of various areas throughout time. The discrepancy between actual and prospective total factor productivities is investigated, as well as the total factor productivity potential growth space after eliminating the resource misallocation component. The following are the key conclusions: the R&D expenditure in this study has a beneficial influence on economic development through TFP, assuming that resource misallocation is ignored. In addition, China's resource misallocation is generally declining, the degree of capital misallocation is decreasing, and labor misallocation is increasing. Among the eight representative industries, the contribution of capital distortion and labor distortion in the eastern region to total factor productivity is −0.036 and 0.065, respectively, which means that the region has sufficient funds, abundant labor force, and high quality, which are followed by the northeast, central, and western regions. It can be seen that the resource allocation efficiency in the eastern region is higher than that in the central and western regions. Market development, trade opening, and industrial structure optimization have significantly reduced the resource mismatch in the eastern region. There are differences in the impact of different factors on resource mismatch between coastal and inland regions. Although the contribution of total factor productivity to economic growth is not very high, partial correlation analysis based on neural network shows that, under the control of the impact of capital and labor input growth on output growth, the correlation coefficient between total factor productivity growth and economic growth is 0.853, which indicates that the growth rate of TFP directly affects the growth rate of GDP [32].

## Figures and Tables

**Figure 1:** Trends in weighted average share of capital income.

**Figure 2:** Output loss from resource misallocation and overall industry misallocation.

**Figure 3:** Simple neuron structure.

**Figure 4:** Threshold function.

**Figure 5:** Linear function.

**Figure 6:** Error curve.

**Figure 7:** Scattered plot of TFP and R&D contribution rate.

**Figure 8:** Contribution of capital distortion and labor distortion to TFP.

**Figure 9:** The impact path of resource misallocation on TFP.

**Figure 10:** Actual TFP and potential growth space for some industries.

**Table 1:** Descriptive statistics for primary variables.

	Valid observations		Mean		Standard deviation	
	2010	2020	2010	2020	2010	2020
Industrial added value	154,183	339,990	21,891	22,110	158,929	171,643
Net value of fixed assets	133,160	303,918	19,615	21,969	107,490	136,513
Number of employees	162,562	304,306	2,891	3,874	20,671	27,079
Account payable	147,726	312,499	14,221	18,203	45,365	53,531
Industrial sales output value	141,675	337,465	25,617	37,657	103,493	120,052

Note: unit means ten thousand yuan/ten thousand people.

**Table 2:** China's total factor productivity measurement results.

Years	TFP	TFP growthrate (%)	Years	TFP	TFP growthrate (%)
2010	0.6984	—	2016	0.8403	−1.83
2011	0.7238	3.64	2017	0.8898	5.88
2012	0.7626	5.36	2018	0.9011	1.27
2013	0.7966	4.45	2019	0.9248	2.64
2014	0.8142	2.22	2020	0.9424	1.90
2015	0.8560	5.13			

**Table 3:** Overall resource misallocation in some Chinese provinces in 2020.

Province	Labor mismatch	Capital mismatch	Province	Labor mismatch	Capital mismatch
Beijing	−0.295	6.522	Jilin province	0.148	−0.456
Henan province	−0.628	0.315	Sichuan province	0.056	0.061
Tianjin	0.299	0.737	Shanghai	0.241	1.035
Hunan province	0.203	−1.600	Jiangsu province	−0.036	1.300
Shanxi province	0.258	0.402	Zhejiang province	0.110	−0.252
Guangdong province	−0.501	0.804	Anhui province	−0.382	−1.152
Liaoning province	−0.055	1.611	Fujian province	0.132	−0.809
Heilongjiang province	0.534	−0.464	Inner Mongolia autonomous region	0.141	−0.241

**Table 4:** Robustness check of resource misallocation delivery mechanism.

Variable	Industrial transfer place		Industry undertaking	
	TFP	Resource misallocation	TFP	Resource misallocation
Lag term	0.012^*∗∗∗*^	−0.115^*∗∗∗*^	−0.09^*∗∗∗*^	0.306^*∗∗∗*^
	(416)	(38.3)	(753.2)	(820.8)

Industrial transfer	−0.043^*∗∗∗*^	−0.348^*∗∗∗*^	−0.336^*∗∗∗*^	−0.357^*∗∗∗*^
	(−2.29)	(−2.77)	(−1.75)	(−1.96)

Resource misallocation	−2.38^*∗∗∗*^	—	−5.59^*∗∗∗*^	—
	(0.22)	—	(−1.89)	—

Control variable	YES	YES	YES	YES

AR (1)	0.444	0.18	0.474	0.182

AR (2)	0.214	0.272	0.373	0.234

## Data Availability

The experimental data can be obtained from the corresponding author upon request.
